# An empirical analysis of the impact of higher education on economic growth: The case of China

**DOI:** 10.3389/fpsyg.2022.959026

**Published:** 2022-08-18

**Authors:** Di Qi, Arshad Ali, Tao Li, Yuan-Chun Chen, Jiachao Tan

**Affiliations:** ^1^Institute of Quality Development Strategy, Wuhan University, Wuhan, China; ^2^Department of Economics and Finance, Greenwich University, Karachi, Pakistan; ^3^School of Economics, Northeast Agricultural University (NEAU), Harbin, China; ^4^School of Foreign Languages and Preschool Education, Beijing Institute of Economics and Management, Beijing, China; ^5^Business School, Zhengzhou University of Industrial Technology, Zhengzhou, China; ^6^The School of Marxism, Central China Normal University, Wuhan, China

**Keywords:** higher education progress, higher education utilization, high-tech industries, economic growth, China

## Abstract

China's domestic labor market has limited demand for tertiary graduates due to an unbalanced industrial structure, with a weak contribution to economic performance over the past decade. This study estimates the asymmetric effects of higher education progress (highly educated employed workforce), higher education utilization (highly educated unemployed workforce), and the separate effects of higher education utilization interactions with high-tech industries on economic growth in China from 1980 to 2020. Using a Nonlinear Autoregressive Distributed Lag (NARDL) model, this study finds that the expansion of higher education progress (the employed workforce with higher education) promotes economic growth, while contraction of higher education progress (employed workforce with higher education) reduces economic growth. Likewise, an increase in higher education utilization (the unemployed labor force with higher education) suppresses economic growth, while a decline in the higher education utilization (the unemployed labor force with higher education) promotes economic growth. The study also found that the expansion of high-tech industries and government spending on education significantly stimulate economic growth. The moderating role of higher education utilization (unemployed labor force with higher education) in the impact of high-tech industries on economic growth is significantly positive. This study strategically proposes that China's higher-educated unemployed labor force can be adjusted to high-tech industries, which need to be developed equally in all regions. Moreover, the country is required to invest more in higher education and the development of high technological industries across all regions, thus may lead to higher economic growth.

## Introduction

Economic theory holds that education, as the main institutional mechanism for the accumulation, production, and diffusion of human capital, is also an externality for the dissemination of market and non-market interests (Schultz, 1961; Becker, 1964; Romer, 1986, 1990; Lucas, 1988). Macro- and microeconomic literature by Acemoglu (2012), Arjun et al. (2020), Campbell and Üngör (2020), Castilla-Polo and Sánchez-Hernández (2020), Fatima et al. (2020), Rico and Cabrer-Borrás (2020), Rossi (2020), Oyinlola and Adedeji (2021), and Braunerhjelm (2022) highlight the importance of education or human capital in the growth process.

Human capital is a complement to Solow's (1956) endogenous growth model, which was augmented by Mankiw et al. (1992). Human capital and technology are directly related to the endogenous growth model proposed by Lucas (1988) and Romer (1990). Economic growth has historically been included in higher education as part of the core mission. A key factor in the growth and technological progress, as the literature has demonstrated, is higher levels of education. The impact of higher education on economic growth has been the focus of scholars over the past two decades. A specialized form of the high level of human capital can be seen as an investment in human capital development.

Asia 2020's strategy is to achieve smart, inclusive, and sustainable growth by putting knowledge at the heart of Asia's efforts (ESCAP, 2020). Linking higher levels of education with research and innovation for personal and social advancement plays a vital role in creating quality human resources, a pressing need for modern technology industries in emerging economies in Asia.

Located on the Pacific coast of Southeast Asia, China is the third largest country in the world after Canada and Russia, with a land area of 9.6 million square kilometers and a population of about 1.35738 billion. China's education system has experienced extraordinary growth and innovation, with the number of students at the higher education level increasing 6-fold from 7.4 million in 2000 to nearly 45 million in 2020, and is considered the largest education system in the world. The country's tertiary gross enrolment ratio (GER) soared from 7.6 to 50%, compared to the current average gross enrolment ratio (GER) in high-income countries of 75%. Currently, Chinese higher education institutions (HEIs) produce 8 million graduates each year, more than the United States and India combined. Needless to say, the democratization of higher education has also been accompanied by an exponential growth in the number of higher education institutions. There are 270 million students at all levels of education in China and 514,000 educational institutions. As one of the most important countries in the world for international education, the speed of China's rise is simply astonishing (Ministry of Education, 2020). According to the statistics of UNESCO (2020), China is the world's largest exporter of international students, and in the 20 years from 1998 to 2017, the number of Chinese students studying abroad for degree programs jumped 590% to more than 900,000. The massive exodus of international students from the world's largest country with a population of 1.4 billion has had an unprecedented impact on global higher education. Large numbers of Chinese students on Western university campuses are a common phenomenon, with three times as many Chinese students registered internationally as students from India, the second largest exporter. Tuition fees and expenses for these students have gradually become a necessary economic factor for local economies and universities in countries such as the UK, the USA, and Canada. About 30% of recorded international students in Australia in 2017 were Chinese. These students help international education become Australia's largest services export, generating nearly $7 billion in onshore revenue.

There are 41.83 million students in 2,738 higher educational institutes (HEIs), including 1,270 undergraduate higher vocational colleges and 1,468 higher vocational education institutions, with a gross enrollment rate of 54.5% in 2020.

The oversight of all higher education institutions (HEIs) in China rests with the Ministry of Education. The mission of the University and Technical University is to lay a high-level theoretical foundation for the nation's incoming scientific workforce. Higher Technical Education Institutions (HTEI) focus more on professional development in scientific and applied research. The higher education system has grown rapidly over the past decade (see Figure 1). The economic returns associated with higher education in China are small compared to other countries, and even during this period the social demand for higher education was high (Bao, 2020; Crawford et al., 2020). Direct low costs and a rising proportion of young people completing secondary education are the main reasons for the increase in demand for higher education (Chen et al., 2019; Pascoe et al., 2020). People determine their higher education, not their employment prospects, but their social status. Also, students can stay as long as they want without worrying about dropping out due to poor grades. Historically, a university degree has been viewed by individuals as a passport into the public sector, offering better working conditions, better pension plans, and higher wages, which have traditionally been preferred over the private sector (Anderson et al., 2020). The demand for higher education is so high that about one in five students in Chinese universities attends overseas universities of the highest caliber in the world (Ma et al., 2021; Xiong et al., 2021). The average years of education of the population, employment, unemployment, and employment with higher education are the human capital stocks that have trended upward over the past 30 years, as shown in Table 1. The average number of education of the employed is lesser than unemployed (Mok, 2016). Kang and Xiong (2021) present a report on empirical evidence that China implements the most significant exception among developed or OECD countries in terms of high unemployment among young graduates. These results indicate that there is a mismatch between the labor market and education, and the domestic economy has limited demand for highly educated talents, while the demand for higher education is strong. Thus, this suggests that the weak link between the labor market and the education system is the main reason for the high unemployment rate of graduates. Latest report highlights China's education insistence without systematic consideration of labor market needs. The domestic economy has limited demand for young tertiary graduates, mainly due to an unbalanced industrial structure that has contributed to the country's poor economic performance over the past decade (Erumban et al., 2019; Chen et al., 2021). As economic activity slumps into these vibrant regions, per capita income and employment are growing faster in coastal regions and other cities than in other provinces. However, areas beyond the coasts are old industrial and energy bases in China's northeastern provinces. The manufacturing industries established in these areas are relatively backward, the economic development is facing major social structural problems, such as unemployment, low living standards, and low per capita income, and energy development has entered a recession period (Chen et al., 2021). The number of university graduates in China is increasing year by year, and the pressure of unemployment has increased dramatically in the past decade. Economic growth slowed from 10.6 to 6.1% in 2010–2020. Hence, to create employment opportunities in technological industrial adjustment, to increase the demand for university graduates, and to achieve economic growth, it is necessary to narrow the gaps in regional industrial structures, establish modern technological industries on an equal footing in all regions, and optimize economic development models.

**Figure 1:** Ministry of education, the people republic of China.

**Table 1:** Average years of education in China, over the period 1980–2020.

**Variables Years**	**1980**	**1990**	**2000**	**2010**	**2020**
Average years of education of Population	6.24	8.29	9.56	11.61	14.12
Average years of education of Employees	6.44	7.99	10.36	11.91	13.26
Average years of education of Unemployed	9.36	10.26	11.29	12.16	14.34
Average years of education of Employees (Higher education)	9%	11%	16%	18%	22%

**Source:** China statistical year book 2020.

This study contributes to the existing literature by empirically examining the asymmetric effects of higher education progress (highly educated employed workforce), and higher education utilization (highly educated unemployed workforce) on economic growth in China using a nonlinear autoregressive distributed lag (NARDL) model, ignoring traditional ARDL model commonly used in other studies. Besides, the study also investigates the effect of higher education utilization (unemployed labor force with higher degrees) in the link between higher technological industry and economic growth in China during the period 1980–2020.

## Literature review

The mature economics literature on the impact of human capital on economic growth underscores Solow's (1956, 1957) early work in neoclassical economics that economic growth can be explained not only by increases in capital and labor but also by technological progress as one of the main factors. Education facilitates the implementation and execution of modern inventive techniques, first proposed by Nelson and Phelps (1966). Countries with large amounts of human capital and lagging technological capabilities may be best placed to catch up with technological leaders faster, in which case productivity gains may be facilitated as human capital levels affect growth. Mankiw et al. (1992) extended the growth model of Solow's (1956) by incorporating an explicit process of human capital accumulation. Incorporating physical and human capital into the Solow model of economic growth determines steady-state per capita income and economic growth. Romer (1986, 1990) proposed a new perspective that extends the theory of endogenous growth by adopting new modern technologies rather than old traditional technologies; his observations reflect that high-skilled labor is an important input required for R&D activities. Such skilled labor is human capital and a key input in the production process. Lucas (1988) believes that education is the carrier and main source of human capital, and an important production input factor in addition to labor and physical capital. This means that a more educated workforce leads to significantly higher levels of productivity, which in turn improves the overall economic outlook.

Higher efficiency productivity and advanced output quality are both possible mechanisms explaining the impact of education on economic growth (Saviotti and Jun, 2020). These two mechanisms can increase the level of purchasing power, thereby stimulating demand and production growth (Matthess and Kunkel, 2020). Although human capital is indeed a key input for accelerating output levels and promoting economic growth. However, measuring human capital remains an important issue. Considering education as the measurement of human capital is displayed in many studies of economic growth literature. However, using education indicators to measure human capital is also divided into multiple dimensions. Four different sets of measures of human capital are (i) enrolment rates, (ii) average years of schooling, (iii) education quality and systems, through international test scores, such as mathematics and science, and (iv) government spending on education as a percentage of GDP (Han and Lee, 2020). Among the four groups of human capital measures given, most empirical studies generally used the average years of education to measure human capital. Habibi and Zabardast (2020) used 18 years of schooling data from 2000 to 2017, applying OLS fixed effects and GMM techniques, to investigate the impact of education on economic growth in the 10 Middle East and 24 OECD countries. The results of the analysis show that education has a positive progressive effect on economic growth in both groups of countries. Another study by Dinh Su and Nguyen (2020) used average years of education as a measure of human capital, using a two-step system GMM estimator, fixed-effects panel quantile regression to investigate the impact of human capital on the economy of 38 African countries from 2002 to 2017. The results of the analysis show that higher accumulation of human capital has a significant positive impact on the economies of African countries. Other studies such as Barro and Lee (2013) and Chen et al. (2019) measure human capital as the average years of education and its positive effect on growth. In addition, many studies looking at enrolment as a proxy for human capital, such as Garza-Rodriguez et al. (2020), applied the method of ordinary least squares to estimate the effect of secondary school enrolment as a measure of human capital on economic growth in Mexico (OLS) during the period 1971–2010. The estimated regression results show that an increase in secondary school enrolment significantly stimulates Mexico's GDP per capita. Another study by Osiobe (2020) used enrolment rates as a measure of human capital and found that human capital had a significant positive effect on economic growth in 14 Latin American countries. Research by Peter Wobst (2005), Pegkas and Tsamadias (2014), Liao et al. (2019), and Hussaini (2020), is consistent with the use of educational enrolment ratios as a proxy for human capital and its possible positive effects on growth.

Uddin et al. (2020) applied the generalized method of moments (GMM) of dynamical systems to a group of 120 developing countries during 1996–2014 to explore the impact of human capital on economic growth. The study found that, as a measure of human capital, investment in education as a percentage of GDP significantly boosted economic growth in developing economies. Similarly, Shafuda and De (2020) also used government spending on education as a proxy for human capital, revealing the positive and significant impact of human capital on Namibia's economic growth over the period 1980–2015. Likewise, Hamdan et al. (2020) and Maneejuk and Yamaka (2021) use education spending as a measure of human capital, which has a significant boost to the Chinese economy. Moreover, Glawe and Wagner (2020) use education quality and systems as measures of human capital, GMM estimates, and the 2003–2007 data period, showing that human capital has a significant positive impact on China's economic growth.

While studies using educational quality and systems as a measure of human capital, such as Glawe and Wagner (2020), using GMM estimates and the 2003–2007 data period, show that institutional quality as a measure of human capital has a significant positive impact on the Chinese economy. Likewise, Agasisti et al. (2021) used GMM estimators to explore the link between the efficiency of the Russian regional higher education system as a proxy for human capital and the speed of regional economic development from 2012 to 2015. The results of the analysis show that the efficiency of higher education institutions has a significant contribution to regional economic growth. Similarly, Agasisti and Bertoletti (2022) also explored the regional higher education system (HES) as a measure of human capital, which had a significant and positive impact on economic growth in 284 European regions over the period 2000–2017. Other studies using high-value education as a proxy for human capital to positively drive economic growth include Martínez-Campillo and Fernández-Santos (2020), Agasisti and Bertoletti (2022).

Several research literatures confirm the positive effects of average years of schooling, enrolment rates, education spending, and education quality on economic growth. However, different education levels have different effects on economic growth, so the further question is: what kind of education level can promote economic growth? Maneejuk and Yamaka (2021) analyzed the impact of primary, secondary, and tertiary education on economic growth in ASEAN-5 for the 2000–2018 data range. The findings show that secondary and tertiary education enrolment rates can boost economic growth in ASEAN-5, but higher education enrolment rates have a greater impact on economic growth than secondary education. Similarly, Bhorat et al. (2016) applied Olley and Pakes' two-stage regression to explore that higher education had no significant effect on economic growth, while education other than higher education had a significant positive effect on the economic growth of the South African economy. Other important studies that prioritize higher education based on strong positive effects on economic growth include Pegkas and Tsamadias (2014), Zhu (2014), Valero and Van Reenen (2019), Habibi and Zabardast (2020), Hamdan et al. (2020), Hussaini (2020), Maneejuk and Yamaka (2021), and Agasisti and Bertoletti (2022).

In general, most of the early studies have demonstrated beyond a doubt the critical role of education in economic growth. Furthermore, many recent studies using various types of datasets and model specifications have considered the strong link between higher education and economic growth. Conversely, some studies argue that higher education investment and university enrollment appear to be less serious than higher education utilization and progress (Alexander, 2020; Blankenberger and Williams, 2020). However, the impact of higher education utilization and progress on economic growth have been rarely studied. Hence, this study considered this gap and decided to fill it by including the workforce with higher education degrees (as a proxy for higher education progress) in our econometric analysis. The study also looked at unemployment at the higher education level, a new measure of higher education utilization. The question of how much the higher education sector contributes to the economy also depends on graduate employment opportunities. Thus, with the increase of highly educated unemployed, the economy will inevitably experience negative growth.

## Model development, data sources, and estimation techniques

### Model development

The aggregate production function of the neoclassical model originally proposed by Solow (1956) is based on the effective pillar, labor, and capital stock. The exogenous factors in the model are technological progress, population growth, and a constant rate of depreciation of capital. Mankiw et al. (1992) augmented the Solow model with human capital and assumed a Cobb-Douglas production function with constant returns to scale and diminishing returns to physical capital and human capital. Mankiw et al. (1992) growth model based on the Cobb-Douglas production function and the Solow growth model is highlighted in the following form:


(1) $$\begin{array}{l} \text{Y}={\text{K}}^{\text{α}}{\text{H}}^{\text{β}}{\left(\text{AL}\right)}^{1-\text{α}-\text{β}} \end{array}$$

where *Y* stands for total production, K indicates physical capital accumulation, H represents human capital, and A and L show technical efficiency and labor, respectively. The model assumes that labor (L) and technical efficiency (A) increase exogenously and at constant rates n and g, respectively. The parameters α and β measure the output elasticity of the relevant input, Transform Equation (1) into a per capita income equation that considers the form of diminishing returns to scale, i.e., α + β < 1.


(2) $$\begin{array}{r} \text{In}\frac{\text{Y}}{\text{L}}=\text{In A}+\text{gt}-\frac{\text{α}+\text{β}}{1-\text{α}-\text{β}}\text{In}\left(\text{n}+\text{g}+\text{λ}\right)\\ +\frac{\text{α}}{1-\text{α}-\text{β}}\text{In}\left({\text{S}}_{\text{k}}\right)+\frac{\text{β}}{1-\text{α}-\text{β}}\text{In }\left({\text{S}}_{\text{h}}\right) \end{array}$$

Where λ represents the depreciation rate of capital, n and g indicate the growth rates of labor and technology, respectively, S_k_ is the investment–output ratio, S_h_ is the investment–human capital ratio, and t shows the time period.

Following the empirical growth model of Mankiw et al. (1992), as mentioned above, the following two econometric models can be derived.


(3) $$\begin{array}{l} \text{Model}:\;1\text{InGD}{\text{P}}_{\text{t}}={\text{α}}_{0}+{\text{α}}_{1}\text{InHE}{\text{P}}_{\text{t}}+{\text{α}}_{2}\text{InHE}{\text{U}}_{\text{t}}+{\text{α}}_{3}\text{InL}{\text{F}}_{\text{t}}\\ \;+{\text{α}}_{3}\text{InCFt}+{\text{α}}_{4}\text{InHT}{\text{I}}_{\text{t}}+{\text{α}}_{5}\text{GEEt}+{\text{ε}}_{\text{t}} \end{array}$$

(4) $$\begin{array}{l} \text{Model}:\;2\text{InGD}{\text{P}}_{\text{t}}={\text{β}}_{0}+{\text{β}}_{1}\text{InHE}{\text{U}}_{\text{t}}^{*}\text{HT}{\text{I}}_{\text{t}}+{\text{β}}_{2}\text{InHE}{\text{U}}_{\text{t}}\\ \;+{\text{β}}_{3}\text{InHT}{\text{I}}_{\text{t}}+{\text{β}}_{4}\text{InHE}{\text{P}}_{\text{t}}+{\text{β}}_{5}\text{InL}{\text{F}}_{\text{t}}\\ \;+{\text{β}}_{6}\text{InC}{\text{F}}_{\text{t}}+{\text{μ}}_{\text{t}} \end{array}$$

GDP is the gross domestic product used as a proxy for economic growth, HEP indicates higher education progress, HEU denotes higher education utilization, LF is the total employed labor force, CF shows capital formation, HTI represents the high-tech industry, GEE is government expenditure on education and ${\text{HEP}}_{\text{t}}^{*}$HTI_t_ illustrate the interaction between higher education utilization and high-tech industry.

### Data sources

Measurements, definitions, and data sources of the variables are explicitly highlighted in Appendix A. The study analysis used annual secondary data for the period 1980–2020.

### Methodology for estimation

A modern approach to the nonlinear autoregressive distributed lag (NARDL) technique introduced by Shin et al. (2014) was used in the study to explore short- and long-term asymmetries in the proposed variables. NARDL methods outperform conventional ARDL procedures in exploring cointegration using small data samples (Amin et al., 2022; Karim et al., 2022). Various studies have used this approach to explore outcome-dependent factors due to the contraction or enhancement of each explanatory factor (Bahmani-Oskooee and Ghodsi, 2017; Syed et al., 2021, 2022; Ullah et al., 2021; Tang et al., 2022).

Following Shin et al.'s (2014) asymmetric cointegration regression


(5) $$\begin{array}{l} {\text{Y}}_{\text{t}}={\text{ρ}}^{+}{\text{e}}_{\text{t}}^{+}+{\text{ρ}}^{-}{\text{e}}_{\text{t}}^{-}+{\text{μ}}_{\text{t}} \end{array}$$

where ρ+ and ρ^−^ are the positive and negative long-term parameters to be estimated. e_t_ is an n × 1 independent factor decomposed into


(6) $$\begin{array}{l} {\text{e}}_{\text{t}}={\text{e}}_{\text{o}}+{\text{e}}_{\text{t}}^{+}+{\text{y}}_{\text{t}} \end{array}$$

The main model of Equation (3) is decomposed into asymmetric Equation (7) by substituting the pessimistic and optimistic sums of Equations (5) and (6).


(7) $$\begin{array}{l} \text{LnGD}{\text{P}}_{\text{t}}={\text{α}}_{0}+{\text{α}}_{1}\text{LnHEP}{\text{t}}^{+}+{\text{α}}_{2}\text{LnHE}{\text{P}}_{\text{t}}^{-}+{\text{α}}_{3}\text{LnHE}{\text{U}}_{\text{t}}^{+}\\ \;+{\text{α}}_{4}{LnHEU}_{\text{t}}^{-}+{\text{α}}_{5}\text{LnLFt}+{\text{α}}_{6}\text{LnCFt}+{\text{α}}_{7}\text{LnGEEt}\\ \;+{\text{α}}_{8}\text{LnHTIt}+{\text{μ}}_{\text{t}} \end{array}$$

The changes of HEP and HEU are decomposed into the sum of their expansion and contraction parts in Equation (7), namely HEP=HEP^+^+HEP^−^, HEU=HEU^+^+HEU^−^, where the plus and minus signs denote HEP and HEU, respectively, expansion and contraction. The partial sums of individual HEP and HEU with positive and negative changes can be derived using the following Equations (8–11).


(8) $$\begin{array}{l} \text{HE}{\text{P}}_{\text{t}}^{+}=\sum_{i=1}^{t}\Delta \text{HE}{\text{P}}_{\text{t}}^{+}+=\sum_{\text{i}=1}^{\text{t}}\text{max}\left(\Delta \text{HE}{\text{P}}_{\text{i}},0\right) \end{array}$$

(9) $$\begin{array}{l} \text{HE}{\text{P}}_{\text{t}}^{-}=\sum_{i=1}^{t}\Delta \text{HE}{\text{P}}_{\text{t}}^{-}+=\sum_{\text{i}=1}^{\text{t}}\text{min}\left(\Delta \text{HE}{\text{P}}_{\text{i}},0\right) \end{array}$$

(10) $$\begin{array}{l} \text{HE}{\text{U}}_{\text{t}}^{+}=\sum_{i=1}^{t}\Delta \text{HEU}{\text{t}}^{+}+=\sum_{\text{i}=1}^{\text{t}}\text{max}\left(\Delta \text{HE}{\text{U}}_{\text{i}},0\right) \end{array}$$

(11) $$\begin{array}{l} \text{HE}{\text{U}}_{\text{t}}^{-}=\sum_{i=1}^{t}\Delta \text{HE}{\text{U}}_{\text{t}}^{-}+=\sum_{\text{i}=1}^{\text{t}}\text{min}\left(\Delta \text{HE}{\text{U}}_{\text{i}},0\right) \end{array}$$

(12) $$\begin{array}{l} \Delta \text{Yt}={\text{α}}_{0}+\text{κ}y_{\text{t}-1}+{\text{κ}}^{+}\text{HE}{\text{P}}_{\text{t}-1}^{+}+{\text{κ}}^{-}\text{HE}{\text{P}}_{\text{t}-1}^{-}+\text{κHE}{\text{P}}_{\text{t}-1}\\ \;+{\text{κ}}^{+}\text{HE}{\text{U}}_{\text{t}-1}^{+}+{\text{κ}}^{-}\text{HE}{\text{U}}_{\text{t}-1}^{-}+\text{κHE}{\text{U}}_{\text{t}-1}+\text{κL}{\text{F}}_{\text{t}-1}\\ \;+{\text{κ}CF}_{\text{t}-1}+\text{κGE}{\text{E}}_{\text{t}-1}+\text{κHT}{\text{I}}_{\text{t}-1}+\sum_{\text{i}=1}^{\text{m}}\beta \text{i}{\text{Y}}_{\text{t}-1}\\ \;+\sum_{i=1}^{m}\text{λ}i\text{HVE}{\text{T}}_{\text{t}-1}+\sum_{\text{i}=1}^{\text{m}}\text{λiL}{\text{F}}_{\text{t}-1}\\ \;+\sum_{i=1}^{m}\text{λ}i\text{C}{\text{F}}_{\text{t}-1}+\sum_{\text{i}=1}^{\text{m}}\text{λiGE}{\text{E}}_{\text{t}-1}\\ \;+\sum_{i=1}^{m}\text{λ}i\text{HT}{\text{I}}_{\text{t}-1}+\sum_{\text{i}=1}^{\text{m}}\text{e}{\text{i}}^{+}\Delta \text{HE}{\text{P}}_{\text{t}-1}^{+}\\ \;+\sum_{i=1}^{m}{ei}^{-}\Delta \text{HE}{\text{P}}_{\text{t}-1}^{-}\sum_{\text{i}=1}^{\text{m}}\text{e}{\text{i}}^{+}\Delta \text{HE}{\text{U}}_{\text{t}-1}^{+}\\ \;+\sum_{i=1}^{m}{ei}^{-}\Delta \text{HE}{\text{U}}_{\text{t}-1}^{-}+{\text{ε}}_{\text{t}} \end{array}$$

Equation (12) above refers to the various steps of the asymmetric ARDL cointegration method.

First, after estimating the null hypothesis Ho = ρ+ = ρ- and the alternative hypothesis H1 = ρ+ ≠ ρ-, the Wald test can be used to explore long-term nonlinear effects. The asymmetric or nonlinear effects of HEP and HEU on economic growth can be determined by accepting alternative hypotheses. κ^+^ and κ ^−^ denote spurs and adverse long-term effects, while $\sum_{i=1}^{k}ui^{+}$ = $\sum_{i=1}^{k}ui^{-}$ or ${\text{u}}_{\text{i}}^{+}$ = ${\text{u}}_{\text{i}}^{-}$ are short-term asymmetric effects of optimistic and pessimistic changes in HEP and HEU.

The asymmetric dynamic multiplier effects of unit changes in ${\text{HEP}}_{\text{t}-1}^{+}$, ${\text{HEP}}_{\text{t}-1}^{-}$, ${\text{HEU}}_{\text{t}-1}^{-}$, and ${\text{HEU}}_{\text{t}-1}^{-}$ are described as follows:


(13) $$\begin{array}{l} M_{\lambda }^{+}=\sum_{i=0}^{k}\frac{\lambda Y_{t+i}}{\lambda HEP_{t+i}} \end{array}$$

(14) $$\begin{array}{l} M_{\lambda }^{-}=\sum_{i=0}^{k}\frac{\lambda Y_{t+i}}{\lambda HEP_{t-i}} \end{array}$$

(15) $$\begin{array}{l} M_{\lambda }^{+}=\sum_{i=0}^{k}\frac{\lambda Y_{t+i}}{\lambda HEU_{t+i}} \end{array}$$

(16) $$\begin{array}{l} M_{\lambda }^{-}=\sum_{i=0}^{k}\frac{\lambda Y_{t+i}}{\lambda HEU_{t-i}} \end{array}$$

Note: M→ ∞, Mp^+^ → α^+^ and Mp^−^ → α^−^, where α^+^ and α^−^ as described above denote long-term asymmetry coefficients. Model stability can be tested using the recursive cumulative sum of residuals (CUSUM) and recursive cumulative residual sum of squares (CUSUMSQ) proposed by Brown et al. (1975).

## Results and interpretation

First, in the empirical analysis, the variables' integration order in the proposed model can be tested using two different unit root tests, Kwiatkowski-Phillips-Schmidt-Shin (KPSS) (Kwiatkowski et al., 1992) and Augmented Dickey-Fuller (ADF) (Dickey and Fuller, 1981). Determining the cointegration relationship among the proposed model variables is based on the level of stationarity of the variables, which will be explored in the first step by unit root tests. Likewise, the ARDL approach cannot be applied with the variables integrated at the second difference, I(2) (Dickey and Fuller, 1981; Kwiatkowski et al., 1992). The KPSS and ADF test results in Table 2 confirm that none of the variables are integrated with the second-order difference I(2), thus validating the use of ARDL techniques in the proposed model. The results in Table 2 show a mix of variable integrations, such as gross domestic product (GDP), higher education progress (HEP), and labor force (LF) at the I(0) level, while capital formation (CF), higher education utilization (HEU), and Government expenditure on education (GEE) are integrated at the first differential I(1).

**Table 2:** Exploring variable integration order with ADF and KPSS testing.

	**ADF**		**KPSS**	
**Variables**	**At level**	**First difference**	**At level**	**First difference**
GDP	−1.546^***^	−2.032^***^	0.435^***^	0.524^***^
HEP	−2.324^***^	−3.256^***^	0.943^**^	0.932^***^
HEU	−3.921	−4.214^***^	0.216	0.421^***^
LF	0.324^***^	1.732^***^	0.423^*^	0.526^***^
CF	−3.25	−4.032^***^	0.352	0.345^***^
GEE	4.456	5.423^***^	0.634	0.824^***^

*, **, and *** are significant levels at 10, 5, and 1%, respectively.

The BDS (Brook et al., 1996) test can be used to detect nonlinear correlations in the presence of a structural break in the data, as shown in previous studies (Manahov and Urquhart, 2021; Selmi et al., 2022). Thus, we can continue to use NARDL after confirming the nonlinear dependencies with the BDS test results in Table 3.

**Table 3:** BDS test for detecting nonlinear dependencies.

**BDS statistics**	**Embedding dimensions = **m****				
	**m = 2**	**m = 3**	**m = 4**	**m = 5**	**m = 6**
GDP	0.2293^***^	0.1296^***^	0.1753^***^	0.2215^***^	0.3242^***^
HEP	0.1462^***^	0.2678^***^	0.3143^***^	0.3245^***^	0.4627^***^
HEU	0.2795^***^	0.2942^***^	0.3256^***^	0.4122^*^	0.4632^**^
LF	0.3236^**^	0.3742^***^	0.2464^**^	0.1632^***^	0.3248^***^
CF	0.1469^***^	0.2136^**^	0.3120^***^	0.1629^**^	0.2167^***^
GEE	0.16293^***^	0.2314^***^	0.3421^***^	0.4971^**^	0.2514^***^

*, **, and *** represent a rejection of 10, 5, and 1% of the null hypothesis, respectively.

Next, the Bound test approach shows that the F-statistic values of 4.994 and 5.898 (highlighted in Table 4) exceed the upper limit of the 1% significance level, indicating that the variables have stable long-term equilibrium relationships.

**Table 4:** Detecting cointegration with Bound testing approach.

	**Model 1**	**Model 2**
F-statistics	4.994^***^	5.898^***^
Lower-upper bound (1%)	3.32–4.48	3.09–4.17
Lower-upper bound (5%)	2.53–3.76	2.29–3.43
Lower-upper bound (10%)	2.23–3.25	2.26–3.31
K	5	5

*, **, and *** are significant levels at 10, 5, and 1%, respectively.

Table 5 shows the long-term variable elasticities results for the NARDL model. Parameter estimation asymmetry can be detected by the sum of the positive and negative parts of HEP_t−1_ and HEU_t−1_, namely ${\text{HEP}}_{\text{t}-1}^{+}$, ${\text{HEP}}_{\text{t}-1}^{-}$, and ${\text{HEU}}_{\text{t}-1}^{+}$ and ${\text{HEU}}_{\text{t}-1}^{-}$ (Bahmani-Oskooee and Nayeri, 2020). The analysis results were very significant for both positive and negative components of HEP_t−1_ and HEU_t−1_. However, different optimistic and unfavorable signs of HEP_t−1_ and HEU_t−1_ have very different effects on economic growth. The stimulation of HEPt-1(HEP+t-1) and HEUt-1(HEU+t-1) coefficients indicated that HEPt-1 significantly promoted long-term economic growth, while HEUt-1 significantly contracted long-term economic growth. The positive coefficient of higher education progress (HEP^+^) is 0.411, indicating that every 1 percentage point increase in higher education progress will significantly boost economic growth by 0.411 percentage points. Likewise, a 1 percentage point contraction in Higher Education Progress (HEP^−^) significantly reduces economic growth by 0.337 percentage points. The findings of this empirical study on the positive and significant impact of higher education progress on economic growth are in good agreement with those of Habibi and Zabardast (2020), Hamdan et al. (2020), Hussaini (2020), Martínez-Campillo and Fernández-Santos (2020), Abad-Segura and González-Zamar (2021), Chentukov et al. (2021), Maneejuk and Yamaka (2021), and Agasisti and Bertoletti (2022). The asymmetric effect of HEPt-1 obviously illustrates that changes in economic growth coincide with increases or decreases in HEPt-1. Likewise, each percentage point increase in higher education utilization (${\text{HEU}}_{\text{t}-1}^{+}$) significantly reduces economic growth by 0.437 percentage points. For every 1% decrease in higher education utilization rate (${\text{HEU}}_{\text{t}-1}^{-}$), long-term economic growth increases significantly by 0.472%. This finding, which argues that a highly educated, unemployed workforce has a detrimental effect on economic growth, is very consistent with research by Ehrlich and Overman (2020), Kim et al. (2020), Zemtsov (2020), and Butkus et al. (2020). The coefficients of high-tech industry (HTIt-1), capital formation (CFt-1), and government education expenditure (GEEt-1) are 0.173, 0.251, and 0.132, respectively, indicating that HTIt-1, CFt-1, and GEEt- increased by 1% can significantly contribute to growth of 0.173, 0.251, and 0.132, respectively. The coefficient of the labor force is also positive but not significant, indicating that the labor force has no significant effect on economic growth. The positive significant coefficient of the interaction term (HEUt-1^*^HTIt-1) in the second model is 0.071, indicating that a 1% expansion of the interaction term can significantly promote economic growth by 0.071%. This means that higher education utilization (unemployed labor force with higher education) has a significant positive moderating effect between high-tech industries and economic growth. This reflects that China's higher level of unemployed labor can be adjusted in high-tech industries, leading to higher growth in the country.

**Table 5:** Long-term variable elasticity results of the NARDL approach.

**Variables**	**Model 1**	**Model 2**
${\text{InHEP}}_{\text{t}-1}^{+}$	0.411^***^ (0.001)	0.642^***^ (0.005)
${\text{InHEP}}_{\text{t}-1}^{-}$	−0.337 (−0.003)	—
${\text{InHEU}}_{\text{t}-1}^{+}$	−0.437^***^ (−0.005)	−0.732^***^ (0.000)
${\text{InHEU}}_{\text{t}-1}^{-}$	0.472^*^ (0.051)	—
InGEE_t−1_	0.132^***^ (0.005)	0.514^**^ (0.033)
InLF_t−1_	0.334 (0.157)	0.464 (0.185)
InCF_t−1_	0.251^***^ (0.004)	0.813^**^ (0.031)
InHTI_t−1_	0.173^***^ (0.002)	0.251^**^ (0.021)
${\text{InHEU}}_{\text{t}-1}^{*}$HTI_t−1_	—	0.071 (0.525)
Constant	−11.723^***^ (0.001)	−9.392^**^ (0.035)
R^2^	0.99	0.91
Adj R^2^	0.81	0.72
F–statistic	623.74	632.89

*, **, and *** are significant levels at 10, 5, and 1%, respectively.

The short-run parameter elasticity analysis in Table 6 shows that changes in economic growth correspond to changes in the partial sum of the positive and negative components of higher education progress (HEPt-1). Such as, the expansion of higher education progress (${\text{HEP}}_{\text{t}-1}^{+}$) significantly boosted economic growth, while the contraction of higher education progress (${\text{HEP}}_{\text{t}-1}^{-}$) significantly reduced economic growth. However, the magnitude coefficient of the sum of the progress part and the unfavorable part (HEUt-1) fluctuates inversely with economic growth, such as the rise of higher education utilization (HEU+t-1) significantly reduces economic growth, while the contraction of higher education utilization (HEU-t-1) significantly promotes economic growth. The moderating effect of higher education utilization (HEUt-1) between high-tech industries and economic growth is positive, but not significant. This means that if the highly educated unemployed labor force adapts to the high-tech industry, it will not be able to drive economic growth in the short term. The coefficients of the error correction term (ECTt-1) of the two proposed models are −0.79 and −0.91, respectively, which are negative and significant, indicating that short-term imbalances can be adjusted to long-term balances ranging from 79 to 91%.

**Table 6:** Asymmetric effects of short-run elasticity of variables in NARDL models.

**Variables**	**Model 1**	**Model 2**
${\text{InHEP}}_{\text{t}-1}^{+}$	0.326^**^ (0.032)	0.437^**^ (0.024)
${\text{InHEP}}_{\text{t}-1}^{-}$	−0.427^*^ (−0.051)	–
${\text{InHEU}}_{\text{t}-1}^{+}$	0.473^*^ (0.071)	0.321^*^ (0.057)
${\text{InHEU}}_{\text{t}-1}^{-}$	0.326^*^ (0.082)	–
InGEEt-1	0.292^**^ (0.031)	0.425^*^ (0.062)
InLFt-1	0.045^**^ (0.012)	0.293^**^ (0.027)
InCFt-1	0.354^***^ (0.002)	0.425^**^ (0.046)
InHTIt-1	0.236^***^ (0.009)	0.724^*^ (0.073)
${\text{InHET}}_{\text{t}-1}^{*}$HTI_t−1_	–	0.216 (0.271)
ECT_t−1_	−0.792^***^ (0.002)	−0.918^***^ (0.000)

*, **, and *** are significant levels at 10, 5, and 1%, respectively.

The models have been checked for heteroscedasticity and autocorrelation issues using diagnostic tests, such as JB, RESET, ARCH, RAMSEY, and LM, as shown in Table 7. This clearly shows that there are no heteroscedasticity and autocorrelation issues in the selected model variables. The variables in the model are not serially correlated, as confirmed by the non-significance of the F statistic used by the Breusch-Godfrey LM test.

**Table 7:** Findings of the diagnostic tests.

**Test**	**Model 1**	**Model 2**
RAMSEY	2.832 (−0.843)	3.934 (−0.432)
JB	2.347 (−0.362)	5.936 (−0.863)
ARCH	1.543(−0.754)	1.325 (−0.436)
RESET	4.769 (−0.874)	8.753 (−0.978)
LM	2.357 (−0.876)	1.874 (0.468)

In parentheses are the respective coefficient probabilities.

The CUSUM and CUSUMSQ tests in Appendices B, C verify the estimated model stability, as the lines in the plots lie within the 5% critical boundary.

Finally, we observe dynamic multipliers to unlock the final growth order dynamics, while accommodating the context of initial differences and short-term dynamics due to unprecedented shocks to higher education progress (HEP_t−1_) and higher education utilization (HEU_t−1_). The existence of such an initial equilibrium is supported by rejecting the null hypothesis in Appendix D, so the validity of the given asymmetric effects highlighted in Table 4 is confirmed by these two plots. Thus, the gradual and significant alignment of economic growth with HEP_t−1_ outflows is dynamic. Optimistic HEPt-1 shocks and unfavorable HEUt-1 shocks are the obvious and most overbearing ones in Appendix D. However, the short-term dynamics take into account the shocks to both economic growth and thus reflect that in all cases, the imbalances are corrected after about 6 years.

## Concluding remarks

This study estimated the dynamic relationship between higher education progress (employed labor force with higher education), higher education utilization (unemployed labor force with higher education), high-tech industries, and other controlling factors and economic growth in China from 1980 to 2020. Besides, the study examines the moderating role of higher education utilization (highly educated unemployed workforce) in the link between high-tech industries and economic growth. This study argues that high-skilled talents produced by higher education can be adjusted in high-tech industries, so China needs to develop high-tech industries equally in all regions. These highly educated workers can significantly contribute to economic growth when employed in high-tech industries.

present study empirically predicts an asymmetric link between HEP_t−1_, HEU_t−1_, and economic growth, whereas the existing literature mainly shows a symmetric link for the specified variables. NARDL results show that the rise of HEP^+^ significantly promotes economic growth, while the contraction of HEP^−^ significantly reduces economic growth. Likewise, the increase in HEU^+^ variation reduces economic growth, and the decline in HEU^−^ volatility significantly stimulates China's long-term economic growth. High-tech industries (HTIt-1) and government spending on education (GEEt-1) have significant positive effects on China's long-term economic growth. The interaction between higher education utilization and high-tech industry (HEPt-1^*^HTIt-1) has gradually contributed significantly to China's long-term economic growth. It can be seen that China's high-tech industries can adjust the high level of China's unemployed labor force, thereby significantly promoting economic growth. Another controlling factor in the model, capital formation, is significant, while the labor force does not significantly drive China's economic growth.

As the above analysis confirms, linking higher levels of education with research and innovation for personal and societal advancement plays a vital role in creating the high-quality human resources that the modern tech industry desperately needs. This high-quality human resource generated by the advancement of higher education can increase productivity levels by employing them in productive sectors such as modern technology industries. Thus, policymakers should place greater emphasis on investment in higher education research and innovation to generate high-quality human resources that meet the needs of high-tech industries. Moreover, this study strategically proposes that as long as China develops high-tech industries equally in all regions, China's highly educated unemployed labor force can adapt to high-tech industries. Hence, the flow of high-quality human resources to the country's high-tech industries can increase productivity levels, thereby boosting economic growth. This strategy is not limited to China, other similar emerging economies such as India, Malaysia, Singapore, and South Korea can also benefit from it to achieve economic transformation.

Regarding study limitations, since this analysis is for a single country, we recommend panel data analysis for future studies to obtain broader conclusions, using the NARDL method for countries with a higher sample.

## Data availability statement

Publicly available datasets were analyzed in this study. This data can be found here: https://datacatalog.worldbank.org/dataset/world~development-indicators.

## Author contributions

JT, TL, and Y-CC conceptualized, revised the study, software, data curation, and literature search. DQ and AA contributed to the conceptualization of the study, analysis, design, conclusions, reviewed the manuscript, and approved the final submission. All authors contributed to the article and approved the submitted version.

## Conflict of interest

The authors declare that the research was conducted in the absence of any commercial or financial relationships that could be construed as a potential conflict of interest.

## Publisher's note

All claims expressed in this article are solely those of the authors and do not necessarily represent those of their affiliated organizations, or those of the publisher, the editors and the reviewers. Any product that may be evaluated in this article, or claim that may be made by its manufacturer, is not guaranteed or endorsed by the publisher.
